The article "Application of Functional Training in Sports Dance Training" was retracted in 2023. Reasons: unreliable results or conclusions; lack of ethics approval or compliance; concerns about the data; concerns about the peer review.

# Application of Functional Training in Sports Dance Training

**DOI:** 10.1155/2022/8695535

**Published:** 2022-08-28

**Authors:** Hualin Ji

**Affiliations:** School of Music and Dance, Xinyang Normal University, Xinyang 464000, Henan, China

## Abstract

With the rapid development of the economy, people's various needs for daily life are also increasing. Because this sport combines sports and dance, which makes the sport have the effect of physical fitness, as well as the emotional edification and visual beauty that dance brings to dancers and audiences. With the increase in people's needs, at the same time, corresponding to the relatively insufficient functional training of the project, this problem makes sports dance, the international standard ballroom dance, always at a low level of development, and at the same time, makes it lack of competitiveness. Also, the nature of dance is now more of a viewing experience. In view of the lack of functional training in international standard ballroom dancing, this article will study the role of functional training in this. By adopting the technology of human body feature recognition and functional action screening, it implements the steps of human action recognition detection technology, human action tracking technology, human body posture shape recognition method, and functional action screening. And the final experimental results show that functional training can screen out 57.3% of female dancers, with ligament damage, and 52.1% of male dancers. The screen outs were more than half of the total numbers, which shows that functional training effectively improves international standard ballroom dance that can provide good assistance for dancers' training.

## 1. Introduction

The vigorous development of the economy has brought people the yearning for a better life, and the sport of sports dance is slowly entering people's field of vision. However, the functional training supporting it has not been developed in time. The international standard ballroom dance evolved from Western social dance, which made the West a leader in this field. They are pushing this sport gradually towards the road of sports competition. For the training of sports dance, the training of dance movements by the dancers themselves can make the beauty of the dance well displayed. This makes most of the audience and even the dancers pay more attention to their own dance techniques, thus ignoring the strengthening of their own functional training. And this problem has greatly restricted the development of China's international standard ballroom dancing, and the characteristics of its own sports competition have not been well developed. It also makes Chinese sports dancers less competitive in international dance competitions. This paper conducts research on the lack of functional training in international standard ballroom dance, in order to improve the comprehensive strength of dancers.

Sports dance training is a very delicate process for professional dancers, and the improvement of dancers' dance skills also depends on the rationality of training. In this regard, many researchers have done a lot of research. Mitrousias et al. studied the dangers of dancing with poles and piles as the background [1]. Liu studied the impact of sports dance on individual students [2]. Dhillon et al. did some cultural research on dance. They conducted specific observational studies on the universality and adaptability of human motion [3]. Purser studied some of the perceptions of dancers of different genders about emotional expression in dance. And he conducted experiments through interviews and also proposed a new dual theory concept to explain the results of his research [4]. Luiggi and Griffet studied the risk of physical exercise and concluded that the physical risk of competitive sports is relatively high, including sports dance [5]. Hanefeld et al. studied the possibility of swing dancing, which can bring happiness to the dancers themselves [6]. The above research and its results are very rich for dance, a big sport, but it has not involved the international standard ballroom dance, which is the sports dance studied in this paper. The mentioned researches more concentrated on the dance movement itself and the influence of dance on people who learn dance, rather than the relevant research on the comprehensive skills of the dancers themselves.

This paper introduces functional training into sports dance, which is to improve the all-round strength of Chinese international standard ballroom dancers. Functional research work has been carried out in recent years. The experiments carried out by Sobrero et al. were intended for research subjects. After a certain functional training, the degree to which the health status of the subjects changes [7]. Lima et al. have shown through experimental research that the elderly will have significantly improved health outcomes after functional training [8]. Lajoso-Silva et al. studied the functional training of firefighters, in which cardiorespiratory function was considered an always important competency [9]. Ko and Lee An conducted research on traditional functional training and establishes a new functional injury prevention normative model on its basis [10]. All the above studies take functional training as a research method, and the targets are different. In general, it has a relatively positive effect in each study. However, the application to sports dance is very less, and the application of functional training to sports competition is also relatively less. In this way, it is difficult to make international standard ballroom dance develop in the direction of sports competition.

This paper studies the application of functional training in international standard ballroom dancing. The purpose of this is to enhance the exquisiteness of the dance movements of the international standard ballroom dance and at the same time strengthen the characteristics of sports competition. In the experiment of functional movement screening, this paper investigates the injury situation of dancers in different dance forms. It can be known from the experiments that the female and male dancers have different types of injuries. Among them, the probability of female ligament injury in modern dance was 57.3%, and for males, muscle injury was 51.2%. The innovations of this paper: (1) this paper shifts the research focus of sports dance from the polishing of dance movements to the functional training of the corresponding dance movements. It provides the basis for the sports competition to realize this project. (2) In the research on the application of functional training in sports dance, this paper adopts two methods of human action feature recognition and functional action screening.

## 2. Application Methods of Functional Training in Sports Dance

### 2.1. Expression Methods of Aesthetic Features of Sports Dance

The emergence of sports dance is the result of the mutual integration of sports competition and dance. Now it has become an international sports event with many fans. This sport has the same fitness function as traditional sports, and at the same time, it also has the characteristics beauty of the posture and the beauty of the dance itself. Moreover, it integrates factors such as music, performance, skills, physical fitness, and aesthetics. Due to its strong ornamental characteristics, it makes most of the audiences and some dancers pay more attention to the dancers' skills. The aesthetic characteristics of different international standard ballroom dance, namely sports dance, are different.

Source and development of sports dance: dance sports, as it is now called, is the result of a gradual formalization through early advocates and enthusiasts. In the early days of this dance movement, it was also known as the international standard ballroom dance. It started from social dance in the West, and with the rise of European countries, it gradually formed a variety of dance projects [11]. In the early days, this type of dance was divided into two categories, and now there are about ten small branches. Its specific classification structure is shown in Figure 1:

Figure 1 above is an explanation of the types of international standard ballroom dance, that is, sports dance. As can be seen from the figure, the dance has 5 dance categories from both Latin dance and modern dance. The production of a series of different dances corresponding to the two is accompanied by the transformation of social dance from nobles to commoners. And because of the characteristics of dance, it can well express the emotions of dancers and audiences. The dance genres described above are based on the development of their origins in the West. After the introduction of sports dance to China, the development of sports dance is slowly in line with the international development. It is also applied in combination with sports competitions, resulting in Chinese-style sports dance.

Aesthetic perspective of sports dance: the meaning of the name of the international standard ballroom dance is the own characteristics of sports dance, that is, “ballroom dance,” which is a dance based on the premise of social interaction. This feature makes the dancers complete the entire dance process by cooperating with each other. As for the beauty displayed by sports dance, there are usually two types, that is, the movement of the dancer's own skills and the artistic content expressed by the dance itself. This is the aesthetic appreciation perspective of traditional dance. But for sports dance, it also has the characteristics of sports competition, with the characteristics of striving for the top spot, which also increases the attraction for the audience. For sports dance, the aesthetic features it contains can be in-depth from the perspective of Figure 2:

Figure 2 above is an overview of the aesthetic perspectives of sports dance. From these aesthetic perspectives, it can be known that the viewing of sports dance can be cut in from many angles. Because of this sport, it combines more intangible things of the dancers involved with the tangible parts such as the movements they show. The combination of human inner and outer makes sports dance contain complex aesthetic characteristics. For the beauty of the figure, it shows the beauty of the dancer's personal health. These include a variety of different comprehensive aesthetic features. This includes manifesting through human form and physical qualities. These include a series of aesthetic elements such as body shape, face, sportswear, posture, line, flexibility, coordination, strength, and so on. For this aesthetic point of view, dancers and dance trainers have different views on the importance of each element in the connotation of body aesthetics. The results are shown in Table 1:

As shown in table, the dancers themselves and the trainers have the aesthetic characteristics of the body shape of sports dance, taking the beauty of the body shape, the beauty of the dance posture and the beauty of the body lines displayed as the important components of the aesthetic point of the sports dance body shape. This is because the physical beauty of sports dance itself is formed by the fusion of the strong and powerful beauty of male dancers and the softness of female dancers [12]. In addition, the dynamic beauty of sports dance is also a major entry point for the aesthetics of dance types studied in this paper. This feature is the comprehensive aesthetic features produced by dancers when performing dance movements. For the same entry point of this aesthetic, dancers and dance trainers have different views on the specific expression of this aesthetic feature. The results are shown in Table 2.

As can be seen from Table 2 above, dancers will pay more attention to the dynamic beauty of the dance itself in dance skills, and the proportion was 72.51%. For dance choreographers and trainers, they will pay more attention to the beauty of the overall dynamic and static combination of dance, and this proportion was 61.75% [13]. The difference in views between the two is due to the fact that the dancers have regarded the technicality of each dance movement as the basis of the dance itself from the beginning of the practice. The trainer's opinion is that it starts from the entire dance process and overall control. In addition, the aesthetic characteristics of the human will also be displayed in the process of dancing. This aesthetic feature is completely developed based on the subjective initiative of the participants, which is often reflected in the dancer's spiritual outlook in dance competitions. For its specific embodiment, the statistical results of the views of dancers and dance trainers are shown in Table 3.

As can be seen from Table 3 above, for dancers participating in the dance movement, they will regard the beauty from the coordination and cooperation between the two participating in the dance as the connotative beauty displayed by the dance. The proportion of dancers who hold this view was 72.69%. For dance trainers, in addition to the above performance as the embodiment of the will aesthetics of the dance, the dancer's deportment aesthetics in the dance will be used as one of the expressions. This is because it pays more attention to a correct attitude displayed by the dancers in the dance. Since the aesthetic characteristics of sports dance are very comprehensive, the aesthetic characteristics displayed by it can roughly include four different directions. The specific entry points are shown in Figure 3.

The aesthetic presentation form of sports dance mentioned in Figure 3 above is only produced by observing the classification of extracted features from some specific angles, and its generalization is high. Among them, the natural properties of tangible materials are like the aesthetic characteristics presented by music, clothing, equipment, and scenes through certain combination rules: neatness, symmetry, balance, rhythm, and diversity. This content includes many external elements, and the aesthetic sense of form is to assemble these things according to certain rules, making the aesthetic sense of viewing more tidier [14].

Functional training methods of sports dance: since the birth of the sports dance project, it has long attached the characteristics of sports competition to the movement. From the psychology of winning the competition at the beginning of the dance to the survival of the fittest reflected in the results of the competition, it is determined that this is not a simple dance sport. Therefore, it is necessary to carry out functional training, which will determine the final result of sports dance dancers. This is the most basic and an extremely important point of sports dance today [15]. Unlike previous training to improve individual dance skills, it will consider the role of functional training more. In the process of sports dance, the dancer is the main bearer of the whole dance. At the same time, dancers will constantly adjust their muscle groups. Therefore, in this process, it is necessary to analyze the corresponding functional consumption of the human body. During exercise of any length of time, the three energy metabolism systems of phosphate, glycolysis, and aerobic oxidation are simultaneously involved in supplying energy every second. It is just that the relative proportions of different phosphogen systems supply energy. At the same time, the glycolysis system is activated, and muscle glycogen is rapidly decomposed for energy supply.  Table 4 is the size of the burden that dancers bear during the dance of various sports dances:

As can be seen from Table 4 above, different dance types have slightly different ways of consuming energy in the dancer's body. And it can also be known that when the function of the dancer's own energy processing organs is poor, the dancer's ability to complete more difficult dance movements will also have a certain impact [16]. Therefore, it is necessary to carry out specific functional training for dancers participating in sports dance competitions. For this training content, it is divided into several parts as shown in Figure 4.

The ten components of functional training are included in Figure 4 above. The most important of these is the strength training for the participating dancers. This is the basic requirement for long-term sports and a major prerequisite for the completion of difficult movements. The second is to have the ability to continuously complete the dance movement from start to finish. The third is the ability to fit the dancer himself, his partner, and the music, and the ability to complete a specified action within a specified time. The above are the components of functional training. To achieve the above content, specific functional training is required [17]. The specific content is shown in Figure 5.

In the above Figure 5, according to the basic part and characteristic part of functional training, the training content is divided into two parts, one is general functional training, and the other is functional training for specific content. The combination of the two is mainly aimed at the strength of the dancer's muscles and the increase in strength in a short period of time, as well as metabolic capacity under aerobic and anaerobic mixed energy supply state, flexibility of each joint, body balance and control ability, coordination ability and sensitivity of body movements, sensitivity to spatial position and direction, and sensitivity to changes in the external environment adaptability, etc., It first strengthens the basic training part, and then performs compound functional training for dance movements [14].

### 2.2. Human Action Recognition Method of Sports Dance

For the research on the application of functional training in sports dance, the mentioned contents are the expected goals of the specific implementation of the training. However, for this series of functional training goals, the most important thing is to use some more effective methods than traditional methods to gradually train in ordinary dance training. This paper intends to adopt the interactive human-machine technology of tracking and recognition in computer science technology. The use of this method is to increase the scientific nature of functional training while ensuring the final result of dance practice [18].

Human motion recognition detection technology: the proposal of this method is based on the mature development of today's computer science and technology. The first introduction is the identification and detection technology. There are usually two methods for human action recognition before this. It usually includes traditional detection techniques and statistical principle detection techniques. Its shortcomings make its application scope narrow. In this paper, the human action recognition detection technology is used in dance training, and new requirements are put forward for the generality of this technology [19]. The implementation of traditional human action recognition detection usually has the following methods. The first is to distinguish the shape of the dynamic object according to the difference between the images of the two consecutive videos, which can be processed by the following formula:

(1) $$\begin{array}{c} X_{a}\left(a,b\right)=\left|f_{u-1}\left(a,b\right)-f_{u}\left(a,b\right)\right|. \end{array}$$

The above operation formula can make the distinction of dynamic objects in the image very good in the case of no external interference. However, because the source of the video is difficult to be guaranteed, noise reduction processing should be performed on the above operation results [20]. The specific processing formula is:

(2) $$\begin{array}{c} \left\{\begin{array}{cc} X_{a}\left(a,b\right)=0, & X_{a}\left(a,b\right)<\lambda ,\\ X_{a}\left(a,b\right)=1, & X_{a}\left(a,b\right)\geq \lambda . \end{array}\right) \end{array}$$

The above formula uses the method of setting the limit value to eliminate the interference caused by the environment and the like. In addition, there are also distinction operations performed on the content in front of a picture and the background of the picture. This method of human action recognition needs to model each image, and the corresponding modeling formula is as follows:

(3) $$\begin{array}{c} Q\left(a,b,c\right)=n\left(a,b,c\right)+m\left(a,b,c\right), \end{array}$$

*Q*(*a*, *b*, *c*) in the above formula is the description expression for the collected pictures, while *n*(*a*, *b*, *c*) and *m*(*a*, *b*, *c*), respectively, represent the dynamic moving objects in the picture and the description for the background of the picture. At the same time, for the dynamic human body that needs to be recognized, the following formula can be obtained through the transformation of the above formula:

(4) $$\begin{array}{c} n\left(a,b,c\right)=Q\left(a,b,c\right)-m\left(a,b,c\right), \end{array}$$

The above operation formula also does not take the interference of the external environment into account. For this, it is necessary to obtain an accurate formula for distinguishing the algorithm through the processing of noise reduction. Its expression is as follows:

(5) $$\begin{array}{c} l\left(a,b,c\right)=Q\left(a,b,c\right)-m\left(a,b,c\right)-x\left(a,b,c\right), \end{array}$$

*l*(*a*, *b*, *c*) in the above formula represents the operational description of the difference between a single image, and *x*(*a*, *b*, *c*) represents the interference information in the environment. In addition, there is a third method, that is, by comparing the projection of the three-dimensional dynamic measured object on the two-dimensional plane and the two-dimensional picture located in the plane. This method is called the streamer method. It then performs corresponding processing on the unidirectional velocities of the two measured objects.

Human motion tracking technology: in order to better collect the action elements of sports dancers, it is necessary to adopt corresponding action tracking technology on the basis of the mentioned human action recognition and detection. The most important thing about this technology is the accurate use of the tracking algorithm. The tracking content of this technology usually includes the tracking of the physical properties of the object to be measured, for the tracking of the lines of the shape of the tested human body, the tracking according to the different proportions of various parts of the human body, and the tracking of the simplified graphics after the abstraction of the human body. This paper will introduce an identifiable technology device with advanced technology [21]. In this way, it can achieve better guidance for sports dance. This device can capture the sound of the collected objects, as well as identify the color of the image, the human body under test and the skeletal structure of the human body. The basic principle is through the encoding process of light and can be represented by Figure 6:

Figure 6 above is a general description of the imaging principle. This process is mainly to collect scattered light spots formed by irradiating the emitted laser on the human body. Based on this, the next step is to collect relevant data for all possible objects in the detected space, and corresponding processing needs to be performed in four steps. It includes calibration, sampling, localization, and reconstruction. The first is to mark specific elements, plus the color of the picture and the information contained in the background, which can express the initial number in the measured space with the following formula. The formula is as follows:

(6) $$\begin{array}{c} l_{r}=P\tan\left(d\cdot l+S\right)-L. \end{array}$$

The *l* in the above formula represents the depth between the coordinates of the original image of the detected point and the background in the space. This formula is used to mark images with different backgrounds. After that, the coordinates of the clear image of the background can be obtained, and the position of each point in the space can also be determined on the coordinates [22]. The corresponding relationship is as follows:

(7) $$\begin{array}{c} \left\{\begin{array}{c} a_{\varepsilon }=\left(a_{l}-\frac{\varepsilon }{2}\right)\cdot \left(c_{\varepsilon }+h\right)\cdot P\cdot \left(\frac{\varepsilon }{d}\right),\\ b_{\varepsilon }=\left(b_{l}-\frac{d}{2}\right)\cdot \left(c_{\varepsilon }+h\right)\cdot P,\\ c_{\varepsilon }=l. \end{array}\right) \end{array}$$

In the above formula, (*a*_*ε*_, *b*_*ε*_, *c*_*ε*_) is the location of the measured point at the background, and (*a*_*l*_, *b*_*l*_, *c*_*l*_) represents the coordinate position of a random point in the measured space. Both *h* and P in the formula are constants. This paper then needs to identify the skeletal structure of the human body accordingly, and in order to define the characteristics of each part of the body, its mathematical expression is as follows:

(8) $$\begin{array}{c} f_{x}\left(\overset{\wedge }{a}\right)\propto \sum_{j=1}^{M}g_{jx}\exp\left(-{\left\|\frac{\overset{\wedge }{a}-\overset{\wedge }{a_{j}}}{y_{c}}\right\|}^{2}\right). \end{array}$$

In the above formula, $\overset{\wedge }{a}$ represents the coordinates of the three-dimensional solid in space, and *M* represents the number of pixels in the collected image. *g*_*jx*_ is the proportion of pixels in the picture, $\overset{\wedge }{a_{j}}$ is the projection of the pixel, and *y*_*c*_ is the width of the feature of the tested human body. This formula can combine the pixels of the image and the human body under test.

### 2.3. Human Posture Morphology Recognition Method and Functional Action Screening

The recognition method for the human body posture is a necessary way to realize the communication between the human and the computer on the posture on the basis of the above detection and tracking. The following introduces several methods for human gesture recognition. The first is human pose recognition known as the Hausdorff distance, two sets of different points, *P*={*x*_1_, *x*_2_,…, *x*_*a*_} and *Q*={*y*_1_, *y*_2_,…, *y*_*b*_}, are assumed, and the Hausdorff distance is used to determine how similar the two sets are. The specific operation process is as follows:

(9) $$\begin{array}{c} H\left(P,Q\right)=\max\left(h\left(P,Q\right),h\left(Q,P\right)\right),\\ h\left(P,Q\right)=\underset{x\in P}{\max}\underset{y\in Q}{\min}\left\|x-y\right\|,h\left(Q,P\right)=\underset{y\in Q}{\max}\underset{x\in P}{\min}\left\|y-x\right\|. \end{array}$$

‖*x* − *y*‖ and ‖*y* − *x*‖ in the above formula represent the Euclidean distance between two point sets, and the operation result obtained by the function represented by *h* is related to the degree of similarity between the two point sets. When the two are more similar, then the Hausdorff distance will be smaller. The calculation of this parameter is also largely disturbed by environmental factors, which can be calculated using a special form of processing formula. The formula is as follows:

(10) $$\begin{array}{c} H_{TK}\left(P,Q\right)=\max\left\{\left(h_{T}\left(P,Q\right),h_{K}\left(Q,P\right)\right\}\right),\\ h_{T}\left(P,Q\right)=T_{x\in P}^{th}d_{Q}\left(x\right),h_{K}\left(Q,P\right)=K_{y\in Q}^{th}d_{P}\left(b\right). \end{array}$$

*T*_*x*∈*P*_^*th*^ in the above formula represents the *T*th point in the *P*-*Q* point set, and *K*_*y*∈*Q*_^*th*^ represents the *K*th point in the *Q*-*P* point set. The above formula will also lose its effectiveness when the environmental interference reaches a certain level. At this time, the average Hausdorff distance can be used for calculation processing. The specific definition formulas are as follows:

(11) $$\begin{array}{c} H\left(P,Q\right)=\max\left(h\left(P,Q\right),h\left(Q,P\right)\right),\\ h\left(P,Q\right)=\frac{1}{r}\sum_{x\in P}\underset{y\in Q}{\min}\left\|x-y\right\|h\left(Q,P\right)=\frac{1}{t}\sum_{y\in Q}\underset{x\in P}{\min}\left\|Q-P\right\|. \end{array}$$

*r* and *t* in the above formula, respectively, represent the number of points in the point set. The second method is the Markov model. This method first assumes that the set of different states in a system under test is *M*={*M*_1_, *M*_2_,…, *M*_*o*_}, and at a certain time *t*, the set of states is *N*^*t*^={*N*_1_, *N*_2_,…, *N*_*t*_}, and at this time, the set of states *M* is in the set of states. The probability of the state occurring can be expressed by the following formula:

(12) $$\begin{array}{c} W\left(N_{t}=M_{i}|N_{t-1}=M_{i},N_{t-2}=M_{k},\ldots \right). \end{array}$$

If the state of the detected human posture at *t* and t–1 is related, a point set in a discretized state can be formed, which can be expressed by the following formula:

(13) $$\begin{array}{c} W\left(N_{t}=M_{i}|N_{t-1}=M_{j},N_{t-2}=M_{k},\ldots \right)=W\left(N_{t}=M_{i}|N_{t-1}=M_{j}\right), \end{array}$$

when only considering the state at time *t*, its formula can be expressed as:

(14) $$\begin{array}{c} W\left(N_{t}=M_{i}|N_{j-1}=M_{j}\right)=q_{ij},\;1\leq j,i\leq o, \end{array}$$

*q*_*ij*_ in the above formula represents the probability of change between different states, and this series of calculations is the method of human gesture recognition. In addition, a method for identification by measuring the angle between human joints was introduced. Assuming that there are two points *A*(*a*_1_, *b*_1_, *c*_1_) and *B*(*a*_2_, *b*_2_, *c*_2_) in the space, the Euclidean distance between them can be expressed by the following formula:

(15) $$\begin{array}{c} d\left(A,B\right)=\sqrt{{\left(a_{1}-a_{2}\right)}^{2}+{\left(b_{1}-b_{2}\right)}^{2}+{\left(c_{1}-c_{2}\right)}^{2}}. \end{array}$$

The calculation of the angle between the joints of the human body can be calculated by the law of cosines, and its formula is as follows:

(16) $$\begin{array}{c} \beta =\;\cos^{-1}\frac{\left(x^{2}-y^{2}+z^{2}\right)}{2xz}, \end{array}$$

*β* in the above formula represents the angle between the two joints, and *x*, y, and *z*, respectively, represent the side length of the triangle where the angle is located. In addition, in order to deal with the error during measurement, the angle between the joints is now defined as:

(17) $$\begin{array}{c} Q=\left\{\left(Q_{1},Q_{2},\beta ,\lambda \right\}\right), \end{array}$$

*Q*_1_ and *Q*_2_ in the above formula represent two different joint points, and *λ* represents the limit value when the included angle is adjusted, when all the changed angles are within this limit value. The pose of the human body as shown in Figure 7 can be recognized.

Figure 7 above is a simple illustration for the recognition of two gestures and angle acquisition. In addition, functional movement screening is also carried out. This method is to collect a large amount of data, and then use certain methods to analyze the movement ability of the human body. The purpose is to better evaluate the standard movements of the athletes participating in the sports. This paper will use the experimental method. The process is shown in Figure 8.

Figure 8 above is the subject of the experiment with dancers in sports dance. It analyzes the possible injury problems of dancers by collecting the relevant data of the tested objects, so as to make a better training plan according to the results of the data.

## 3. Application Experiment and Result Analysis

### 3.1. Investigation Experiment and Result of Aesthetic Characteristics of Sports Dance

For the study of the aesthetic characteristics of sports dance, this paper has carried out relevant analysis from multiple perspectives in the previous method section and collected the opinions of dancers and dance trainers accordingly. In addition, the influence of the background music of the dance on the dancer's alternate steps during the dance is also needed here, and this directly affects the dancer's dance process. For a professional sports dancer, the control of the dance pace and rhythm is very flexible. Based on the music background, they also need to adjust themselves.  Table 5 shows the comparison results of the beats of several sports dances in different periods:

As can be seen from Table 5 above, with the development of sports dance, dancers' grasp of dance rhythm has undergone relatively subtle changes. That is, in the twentieth century, various dances were usually defaulted to have only one rhythm, and the number of beats was as many as the number of steps. But today's sports dance will add a few steps on the original basis, and this result can improve the overall beauty. The Viennese waltz in the table is the fastest dance, now reaching 61 beats a minute. The prevalence of this dance now also illustrates this point. And it also shows that the tempo of the music has slowed down. This also emphasizes that the musical duration of the dance steps must be extended, and the compound rhythm provides more possibilities for changing the speed of the movements. In addition, there are people's perceptions of different aesthetic characteristics of dance, and the survey results are shown in Table 6.

From Table 6 above, it can be seen that for the dancers themselves, the most important aesthetic feature is the edification nature of the dance itself to the audience. At the same time, dance trainers also support this view, with support rates reaching 73.15% and 51.39%, respectively. However, the support rate for the feature of expressing emotion in dance is the lowest in these two perspectives. This also shows that the current dancers and their trainers do not have a clear control of this feature. In addition, the specific content of dance training is different, and it also shows different importance. The entry point for this level of importance can be from two perspectives. One is the category of physical actions and the specific performance of actions. The specific results are shown in Figure 9:

From Figure 9 above, it can be seen that the basic movements in the dance shape training project are very important and the highest. It finally reached 72%, which is consistent with the previous results, indicating that the basic skills of dance have a high status in the entire dance training. In the action category, the requirements for the strength of individual dancers are quite high, reaching 87.5%. It is proved that the functional training of this paper is very necessary. In addition, the influence of the dancer's inner state on the presentation effect of the dance is also studied, and the psychological state is also divided into two categories. One is the dancer's own characteristics, and the other is the psychological state displayed by the dancer's dance. The results are shown in Figure 10:

As can be seen from the above Figure 10, the subjects under investigation regard the aesthetic awareness of dance as the most important psychological state in the dance process. Then, there is the level of self-confidence of the dancer, which is less important for the psychological control of the audience, which shows that the dancer has high requirements for himself.

### 3.2. Human Action Recognition Experiment of Sports Dance and Results

The experiments here are based on the application of human action detection and recognition and human action tracking technology constructed in the previous article. In this paper, the angle changes between the detected joints of the specific parts of the limbs of the dancers are recorded during the dance. It then collects the corresponding data of the dancer through the use of the above two technical equipment, and then compares the difference between the two through calculation. The purpose is to train trainers at different levels according to their own level. The results are shown in Figure 11:

From the upper left picture in Figure 11 above, it can be seen that the angle formed by the three joints of the dancer's wrist-elbow-shoulder is relatively large. It hits 108.5, and the waist-knee-ankle angle is also huge at 153.1. This series of comparisons can provide relevant guidance for dancers' training. The dotted line in the figure is the standard angle between joints set by the device. It can finally make the dancer's dance state reach a better state.

### 3.3. Experiment and Result of Functional Movement Screening

The main purpose of this paper is to realize the application of functional movement screening in sports dance. One is to adjust the dancer's dance movements, and the other is to analyze the most likely injuries in the dance. And this has two purposes. For this experiment, we first investigate the types of injuries that may occur in dance through a study of injuries in two sports dance dancers. The specific results are shown in Figure 12.

From Figure 12(a) in Figure 12 above, it can be seen that female dancers have a higher probability of being scratched in their self-love dance. The number of injuries accounted for 43 people, which is also the most important type of injury among male dancers, reaching 23 people. In the modern dance, female dancers are the most vulnerable to ligament damage, while men are to muscle damage. The former accounts for 57.3% of the population and the latter accounts for 52.1%. The reason for the appearance of the former is that women play a major role in Latin dance and need to undertake a large number of dance movements and skills. In addition, frequent muscle control during competition and training, muscle stretching is very easy to cause muscle strain, and the probability of joint dislocation and fracture during competition training are very low.

## 4. Conclusion

This article is a discussion on the application of functional training in sports dance. It makes the dancers themselves need to change from focusing only on the technique of dance and ignoring the function of dance moves to improving their comprehensive strength. This paper firstly applied human body gesture recognition to provide scientific guidance to dancers' dance, and then self-love introduced functional movement screening to investigate the possibility of injury in dance. The research in this paper will be beneficial to the improvement of dancers' comprehensive strength in dance techniques, because the research in this paper provides a more scientific guidance method, that is, a guidance method based on human action recognition. This will bring new opportunities for the development of sports dance.

## Figures and Tables

**Figure 1:** Category branch diagram of sports dance.

**Figure 2:** The connotation of the aesthetic perspective of sports dance.

**Figure 3:** Aesthetic form of sports dance.

**Figure 4:** Functional training composition of sports dance.

**Figure 5:** Specific methods of functional training.

**Figure 6:** Schematic diagram of human tracking device imaging.

**Figure 7:** Angle differences between joints in different poses.

**Figure 8:** Trial flow chart for functional motor screening.

**Figure 9:** Survey results on the importance of dance training content. (a) The results of the importance of body types. (b) Action class importance results.

**Figure 10:** The importance of mental state in sports dance. (a) The dancer's own characteristics. (b) The mental state of the dancer when dancing.

**Figure 11:** Comparison of the joint angles of the three movements of the trainer.

**Figure 12:** Sports dance injuries. (a) Injuries in Latin dance (b) Injuries in modern dance.

**Table 1:** Results of dancers' and trainers' perceptions of aesthetic elements of body shape.

	Sports dancer		Sports dance instructor	
	Frequency	Percentage	Frequency	Percentage
Aesthetic content	110	60.15	17	61.52
Body beauty	68	37.48	7	18.76
Beauty	62	35.16	5	21.45
Beauty of clothing	82	46.78	8	56.17
Posture beauty	115	66.15	18	39.15
Beautiful lines	45	24.57	10	26.13
Flexible beauty	58	31.15	8	31.32
Coordinating beauty	45	24.51	7	22.41
Beauty of strength	0	0	0	0

**Table 2:** Results of dancers' and trainers' perceptions of dynamic aesthetic performance.

Aesthetic content	Sports dancer		Sports dance instructor	
	Frequency	Percentage	Frequency	Percentage
Dynamic and still beauty	121	68.19	18	61.75
Style beauty	65	35.17	10	35.12
Innovative beauty	87	53.12	15	58.17
Beautiful rhythm	85	48.68	13	47.15
The beauty of technology	126	72.51	8	28.51
Other	0	0	0	0

**Table 3:** Results of dancers' and trainers' perceptions of volitional aesthetic performance.

Aesthetic content will beauty	Sports dancer		Sports dance instructor	
	Frequency	Percentage	Frequency	Percentage
Etiquette beauty	85	47.15	15	47.11
Moral beauty	91	54.12	16	51.21
Graceful	55	32.15	7	25.18
Beautiful quality.	76	46.16	10	38.19
Collaborative beauty	57	34.15	6	26.15
Self-cultivation	126	72.69	13	54.15
Other	46	27.85	5	22.43
Aesthetic content	0	0	0	0

**Table 4:** Ratio of energy burden to dancers during sports dance.

Kind of dance		Below 160 bpm	160–169 bpm	170–1 79 bpm	Above 180 bpm
Standard dance	Waltz	47.71	41.12	13.12	0
	Tango	25.31	24.13	32.15	16.8
	Vienna waltz	22.15	14.51	9.15	33.13
	Foxtrot	37.15	45.13	35.15	6.72
	Quickstep	18.61	12.31	47.16	31.79

Latin dance	Rumba	21.71	31.18	13.25	0
	Precisely	18.52	7.61	15.17	62.13
	Samba	18.65	11.55	16.78	49.15
	Bullfighting	25.11	13.12	21.23	35.68
	Cowboy	15.7	6.75	9.8	67.31

**Table 5:** Comparison of beats of sports dances in 9 different periods.

Dance events	2zero century music (bar/min)	Current music (bars/min)
Waltz	31	28∼32
Tango	35	30∼33
Trot dance	61	51∼53
Foxtrot dance	33	27∼30
Vienna waltz	61	59∼61
Rumba	57	24∼28
Cha cha cha	47	31∼35
Cowboy dance	48	42∼45
Samba dance	53	51∼52

**Table 6:** Aesthetic properties of sports dance.

Aesthetic characteristics of sports dance	Sports dancer		Sports dance instructor	
Normative	Frequency	Percentage	Frequency	Percentage
Infectivity	85	51.25	11	34.17
Lyricism	126	73.15	16	51.39
International	47	27.61	7	22.16
Figurative	80	46.15	17	58.15
Diversity	105	61.17	8	31.14
Rhythm	91	52.18	8	31.14
Other	0	0	0	0

## Data Availability

The data used to support the findings of this study are available from the author upon request.
